# Long noncoding RNA ZFAS1 promotes tumorigenesis and metastasis in nasopharyngeal carcinoma by sponging miR‐892b to up‐regulate LPAR1 expression

This article has been retracted.

**DOI:** 10.1111/jcmm.14823

**Published:** 2019-12-18

**Authors:** Jiaojiao Peng, Feng Liu, Hong Zheng, Qi Wu, Shixi Liu

**Affiliations:** ^1^ Department of Otolaryngology, Head and Neck Surgery West China Hospital Sichuan University Chengdu China

**Keywords:** long noncoding RNAs, *LPAR1*, miR‐892b, nasopharyngeal carcinoma, ZFAS1

## Abstract

**Objective:**

In this study, we explored the NPC‐specific expression of ZFAS1 and the mechanism of ZFAS1‐mediated growth, aggressiveness and tumorigenesis in NPC.

**Methods:**

The expression profile of lncRNAs was detected in NPC tissues and matching para‐carcinoma tissues using microarray analysis. LncRNA‐miRNA and miRNA‐mRNA interaction networks were constructed using the miRcode v11 and TargetScanHuman v7.2 web server and then validated using dual‐luciferase assay. Western blot and RT‐qPCR were performed to detect protein and RNA expression. The effects of ZFAS1, miR‐892b and LPAR1 dysregulation on the proliferative, migratory and invasive abilities of NPC cells were observed using colony formation, cell counting kit‐8 (CCK‐8) and transwell assays in vitro. In vivo, a xenograft nude mouse model was established to detect the impact of ZFAS1 dysregulation on the tumorigenicity of NPC cells.

**Results:**

The expression of multiple lncRNAs, of which ZFAS1 was up‐regulated, was dysregulated in NPC tissues. ZFAS1 directly targeted miR‐892b, and miR‐892b negatively regulated the expression of downstream LPAR1. The proliferation, migration and invasion of NPC cells could be largely enhanced by the downregulation of miR‐892b as well as the up‐regulation of ZFAS1 and LPAR1, while the overexpression of miR‐892b and the downregulation of ZFAS1 and LPAR1 decreased these abilities. In nude mice, the growth of tumour xenografts formed by HONE1 cells was significantly suppressed when ZFAS1 was silenced.

**Conclusion:**

The study demonstrated that lncRNA ZFAS1 may act as a promoter of tumorigenesis and metastasis in nasopharyngeal carcinoma, by up‐regulating the expression of LPAR1 in a miR‐892b‐dependent manner.

## 1 INTRODUCTION

Nasopharyngeal carcinoma (NPC) is a common epithelial malignancy of the head and neck, which is prevalent mainly in Southeast Asia, North Africa and Southern China.^1^, ^2^ In these endemic regions, the incidence rate of NPC can reach 15‐50 per 100 000 population.^3^ Due to the high sensitivity to irradiation and surgical constraints, radiotherapy has been the most promising and efficient treatment for the early stage NPC.^4^ However, the survival of patients with advanced NPC is still unsatisfactory, although other adjuvant therapies such as chemotherapy have been performed.^5^, ^6^ On the other hand, late toxicities, including xerostomia, trismus and temporal lobe neuropathy (TLN), are inevitable, and these side effects severely impair the functional status and quality of life of patients.^7^ Therefore, understanding the molecular mechanism of NPC may provide a new direction for diagnosis and treatment.

Recent studies suggest that non‐protein‐coding RNAs (ncRNAs) account for a large proportion (more than 98%) of genome encoded‐transcripts.^8^ Decreased expression of ncRNAs, especially lncRNAs (larger than 200 nucleotides) and microRNAs (miRNAs, 19 ~ 22 nucleotides), has been implicated in the progression of various diseases including cancer.^9^, ^10^ Recently, increasing evidence has demonstrated that lncRNAs can mediate the progression of tumorigenesis and metastasis in a variety of cancers by dysregulating gene expression at the transcriptional, post‐transcriptional or epigenetic level.^11^ Aberrant expression of lncRNAs has also been involved in the initiation and progression of NPC, as reported by several previous studies.^12^, ^13^, ^14^ For example, the expression of lncRNA ANRIL is significantly elevated in NPC tissues, which has been negatively associated with the overall survival of patients, and ANRIL silencing by specific shRNA can effectively inhibit the proliferation and tumorigenesis of NPC cells.^15^ Another study by Li, *et al* 16 also demonstrated the dysregulation of lncRNAs, which markedly mediated the progression of NPC, because lncRNA‐ROR largely promoted proliferation and metastasis through the suppression of the p53 signalling pathway. ZFAS1 is a newly identified lncRNA that is up‐regulated in several human cancers, such as gastric cancer,^17^ non‐small cell lung cancer 18 and hepatocellular carcinoma.^19^ Although the latest encouraging research has reported that up‐regulated ZFAS1 acts as a promoter for the occurrence of NPC through the activation of the Wnt/β‐catenin pathway, the role of ZFAS1 in NPC requires further investigation.^20^

MiRNAs, a group of short noncoding RNAs, bind to target mRNAs by incomplete complementarity and then inhibit the translation or reduce the stability of target mRNAs.^21^, ^22^, ^23^ Multiple miRNAs including miR‐1, miR‐let‐7 and miR‐138 participate in the tumorigenesis, progression and metastasis of NPC through biological functions, such as inducing apoptosis and inhibiting proliferation. Recently, miR‐892b has been found to be associated with bladder cancer 24 and breast cancer.^25^ Particularly, decreased expression of miR‐892b in the plasma of NPC patients has been reported, and miR‐892b expression was up‐regulated after treatment with radiotherapy or chemotherapy.^26^ Thus, miR‐892b may act as a crucial tumour suppressor for NPC, and its roles in the progression of NPC deserve an in‐depth investigation.

As non‐protein‐coding RNAs, miRNAs play a role in various diseases by regulating the expression of genes mainly at the post‐transcriptional level. Here, we identified that the downstream effector of miR‐892b is lysophosphatidic acid receptor 1 (LPAR1). LPAR1, also known as endothelial differentiation gene 2 (EDG2), is widely expressed in various organs to mediate diverse biological functions, including the proliferation, chemotaxis and invasion of tumour cells.^27^, ^28^ Recent studies have found that LPAR1 is a carcinogenic factor and able to enhance metastasis and invasion in several cancers, such as melanoma, breast cancer and ovarian cancer.^27^, ^29^, ^30^ However, to the best of our knowledge, the expression characteristics of LPAR1 in NPC patients as well as the relationship between low expression of LPAR1 and NPC development are still unknown.

In this study, we determined the expression profile of lncRNAs in NPC tissues to emphatically analyse the functions of up‐regulated ZFAS1 and the underlying mechanism. Then, we identified ZFAS1 targeted miRNA (miR‐892b) and the downstream effector protein (LPAR1). The effects of the dysregulation of ZFAS1, miR‐892b and LPAR1 separately on the proliferative, migratory and invasive abilities of NPC cells were detected. In conclusion, our present studies demonstrate that the overexpression of ZFAS1 can aggravate NPC progression through sponging miR‐892b to promote the expression of downstream LPAR1.

## 2 MATERIALS AND METHODS

### 2.1 Clinical samples

NPC tumour tissues and matching para‐carcinoma tissues were collected from 53 patients who had signed an informed consent form, and the clinicopathological features of participants were listed in Table S1. The recruited subjects had no medical history of other malignant tumours and had never undergone any preoperative treatment including chemotherapy or radiotherapy. Sample collection and usage were approved by the West China Hospital, Sichuan University.

### 2.2 Cell culture

The human nasopharyngeal epithelial cell line NP69 and NPC cell lines (HONE1, CNE, HNE1 and C666‐1) were commercially obtained from BeNa Culture Collection (Beijing, China). NP69 cells were maintained in serum‐free keratinocyte medium containing 0.2 ng/mL human recombinant epidermal growth factor, 2% heat‐inactivated foetal bovine serum (FBS), 40 μg/mL bovine pituitary extract and 1% streptomycin and penicillin (Invitrogen, Carlsbad, CA, USA). CNE, HNE1 and C666‐1 cells were maintained in 90% RPMI‐1640 medium containing 10% FBS, and 1% streptomycin and penicillin. HONE1 cells were maintained in DMEM medium containing 5% FBS, 5% newborn calf serum and 1% streptomycin and penicillin. After incubation for 36 hours, cells were harvested to extract total RNA, and then real‐time RT‐PCR (qRT‐PCR) was carried out as mentioned below. Due to the highest expression level of ZFAS1 compared with other NPC cells, the HONE1 cell line was selected for the subsequent cell‐based experiments.

### 2.3 LncRNA microarray analysis

Total RNA was extracted from fresh‐frozen NPC and matching para‐carcinoma tissues using the TRIzol reagent (Invitrogen) according to the manufacturer's protocol. The concentration and purity of the isolated RNA samples were determined using a Nano‐200 spectrophotometer (Aosheng, Hangzhou, China). To identify the lncRNA profiles associated with nasopharyngeal carcinoma, five paired NPC tumour tissues and matching para‐carcinoma tissues were provided to KangChen Bio‐tech (Shanghai, China). Briefly, RNA was labelled using an Arraystar Super RNA Labelling Kit, and then the labelled lncRNAs were hybridized onto an Arraystar Human LncRNA Microarray V4.0 (Arraystar, Rockville, MD, USA), which contained 40173 lncRNAs. The data were analysed with a Robust Multichip Analysis algorithm using the Affymetrix default analysis settings with global scaling as the normalization method. To determine the significance of the differences and the false discovery rate (FDR), thresholds of *P* < .05 and FDR < 0.05 were used. Gene expression fold changes of either >2 or <0.5 were set as the default filter criteria for identifying significantly differentially expressed genes.

### 2.4 RNA reverse transcription and quantitative real‐time PCR

To synthesize cDNA, total RNA was reverse transcribed using a PrimeScript RT Reagent Kit (Takara, Japan) and a miRNA qPCR Quantitation Kit (GenePharma, Shanghai, China) according to the manufacturers’ instructions. Real‐time PCR was carried out as described by the manufacture using PowerUp^TM^ SYBR^®^ Green mixture (Thermo Fisher Scientific, Waltham, MA, USA). Primers were listed in Table S2. Quantification of ZFAS1 and LAPR1 expression was normalized to GAPDH expression, and miR‐892b expression was normalized to U6 expression using the 2‐^ΔΔCt^ method. Additionally, all samples were run in triplicate.

### 2.5 Cell transfection

The ZFAS1 overexpression vector (pcDNA3.1‐ZFAS1, p‐ZFAS1), ZFAS1‐targeting siRNA (siZFAS1), ZFAS1‐targeting shRNA (shZFAS1), miR‐892b mimics or inhibitor and LPAR1‐targeting siRNA (siLPAR1) were commercially provided by GenePharma, and the sequences of siZFAS1 and siLPAR1 are listed in Table S3. Because siRNA is transiently expressed in cells and shRNA can be stabilized by viral‐mediated transduction, in this study, siRNAs were used to knock down expression in vitro, while shRNAs were used in vivo. HONE1 cells were seeded into 12‐well plates (Corning Incorporated, Corning, NY, USA) and transfected by Lipofectamine 2000 following the instructions of manufacturer (Invitrogen). Empty pcDNA3.1 vector, mimics control and non‐targeting siRNAs (siNC) were used as negative controls.

### 2.6 Cell proliferation, migration and invasion assays

Cell proliferation was evaluated using CCK‐8 and colony formation as previously described.^31^, ^32^ For the CCK8 assay, 1 × 10^4^ cells were grown in 96‐well plates in which CCK‐8 reagent was added according to the standard protocol (Beyotime, Beijing, China). Subsequently, the absorbance at 450 nm was measured by a platereader (Thermo Fisher Scientific). For colony formation assay, approximately 200 cells were grown in 6‐well plates for 2 weeks. Then, the cells were fixed with ethanol and stained with 0.1% crystal violet (Solarbio, Beijing, China).

According to a published procedure, the invasive and migratory abilities of HONE1 cells were evaluated with a transwell assay.^33^, ^34^ Cells in the bottom chamber were stained using crystal violet and counted under an optical microscope.

### 2.7 Dual‐luciferase reporter assay

LncRNA‐miRNA and miRNA‐mRNA interaction networks were established using the miRcode v11 (http://www.mircode.org/) and TargetScanHuman v7.2 (http://www.targetscan.org/) web server. MiR‐892b was selected as a promising target of ZFAS1, and its downstream target is LPAR1. A dual‐luciferase assay was carried out to verify the predicted relationships between ZFAS1 and miR‐892b as well as miR‐892b and LPAR1. Luciferase reporters containing the wild‐type 3’‐UTRs of ZFAS1 and LPAR1 (which contain the predicted binding site of miR‐892b) or mutant 3’‐UTRs of ZFAS1 and LPAR1 (the predicted binding site of miR‐892b was mutated) were constructed by Sangon‐Biotech (Shanghai China). Specifically, fragments containing miR‐892b‐binding site‐1 (nucleotide region from 440 to 846) and site‐2 (nucleotide region from 1137 to 1609) in LPAR1 3’‐UTR were cloned into two reporter vectors. MiR‐892b mimics or scrambled oligonucleotides (mimics‐control) were commercially provided by GenePharma (Shanghai, China). The constructed reporters were cotransfected into 293T cells with *Renilla* reporters and miR‐892b mimics or mimics‐control. For luciferase assay performed in HEK‐293T cells, cells in 24‐well plates were cotransfected with 200 ng/well luciferase reporter constructs, 400 ng/well miR‐892b mimic or mimic control using Lipofectamine 2000. In this assay, 5 ng/well SV‐*Renilla* luciferase plasmid served as the internal control. Cells were harvested 24 hours after transfection, and luciferase activity was detected using the Dual Luciferase Reporter Assay kit (Promega) according to the manufacturer's instructions. Firefly luciferase activities were normalized to *Renilla* luciferase activity.

### 2.8 Xenograft mouse model

Four‐week‐old male BALB/c nude mice (n = 20) were commercially provided by Cavens Laboratory Animal Co., Ltd. (Beijing, China). Animals were maintained in a pathogen‐free environment with controlled temperature (22 ± 1°C) and circadian rhythm (12 hours dark/light cycles). HONE1 cells (1 × 10^6^) with stable transfection of shZFAS1 or p‐ZFAS1 were subcutaneously implanted into the back area (4 mice per group). The length and width of tumour xenografts were measured using calipers every 7 days, while the tumour volume was calculated by the following formula: tumour volume = 0.5 × length × width × width. After 21 days, all animals were killed, and tumour xenografts were harvested, imaged and weighed. The expression of ZFAS1 in tumour xenografts was measured using qRT‐PCR.

### 2.9 Western blot analysis

The expression of LPAR1 in HONE1 cells was also evaluated at the protein level by Western blot. In brief, after 72 hours of incubation, HONE1 cells were harvested, trypsinized, washed and lysed in 1× cold RIPA buffer (Beyotime). Protein lysates were quantified, electrophoresed and transferred onto PVDF membranes (Merck Millipore, Billerica, MA, USA). Membranes were blocked with 5% nonfat milk at 37°C for 1.5 hours, followed by incubation with an antibody against LPAR1 (1:2000 dilution, Santa Cruz Biotechnology, Santa Cruz, CA, USA) for 1.5 hours. After incubation with HRP‐conjugated secondary antibody, protein bands were visualized using an ECL detection kit (Amersham Biosciences, Buckinghamshire, UK).

### 2.10 Statistical analysis

In vivo data are expressed as the mean ± SEM, and ex vivo data are expressed as the mean ± SD. Statistical analysis was performed within GraphPad Prism 6.0 (GraphPad Software Inc). Analysis of statistically significant Difference was conducted by t test between two sets of data. For three groups or above, one‐way ANOVA with repeated measures followed by Tukey's post‐tests and two‐way ANOVA with repeated measures followed by Bonferroni post‐tests were adopted. Differences with *P* < .05 were considered statistically significant.

## 3 RESULTS

### 3.1 Expression of ZFAS1 in NPC tissues and cells

The overall pattern of lncRNA expression in NPC tumour tissues was determined using microarray analysis, which was generated for five NPC tumour tissues and their matching para‐carcinoma tissues. Under the conditions of *P*‐value < .05 and fold‐change value >2, six up‐regulated as well as fourteen down‐regulated lncRNAs were identified, of which ZFAS1 was up‐regulated (Figure 1A). The six up‐regulated lncRNAs were verified in a larger sample size (n = 53) by qRT‐PCR, and the results showed that ZFAS1 expression was truly and significantly up‐regulated in NPC tissues compared with noncancerous para‐carcinoma tissues. Among the six identified lncRNAs, ZFAS1 appeared to have the highest fold change in 53 NPC tumour tissues (*P* < .01, Figure 1B). Based on the expression level of ZFAS1, patients were assigned into low‐expression and high‐expression groups. Then, an analysis of the relationship between ZFAS1 expression and the clinical parameters of patients including gender, age, tumour stage and relapse were performed (Table S1). The results showed that the expression level of ZFAS1 was positively associated with clinical T stage (*P* = .0281) and TNM stage (*P* = .0281) in NPC patients, while associations with gender (*P* = .7846), age (*P* = .3520), histological classification (*P* = .7570) or relapse (*P* = .1757) were not significant. Compared with expression in the noncancerous NP69 cells, ZFAS1 was also obviously up‐regulated in the NPC cell lines including HONE1, CNE, HNE1 and C666‐1 (*P* < .05, Figure 1C). Interestingly, the expression of ZFAS1 was altered in different NPC cells, and HONE1 cells presented the highest expression compared with other NPC cell lines. Therefore, HONE1 cells were selected for the subsequent cell‐based experiments.

**Figure 1:** Upregulation of lncRNA ZFAS1 in NPC tissues and cells. A, Profile of differentially expressed lncRNAs in normal (n = 5) and NPC tissues (n = 5). Twenty representatives lncRNAs with the most‐significant changes are plotted, and the up‐regulated lncRNAs are coloured with purple, and the down‐regulated lncRNAs are coloured with brown. ZFAS1 was up‐regulated. B, The levels of six up‐regulated lncRNAs were further detected in 53 NPC tumour tissues and matching para‐carcinoma tissues and ZFAS1 showed the highest fold change (n = 53). **P < .01. C, Expression of ZFAS1 was up‐regulated in various NPC cell lines compared with human noncancerous nasopharyngeal epithelial cell line (NP69 cells). *P < .05 and **P < .01 compared with NP69 cells

### 3.2 ZFAS1 positively affects the proliferative, migratory and invasive abilities of HONE1 cells **in vitro**

The effects of transfection with p‐ZFAS1 and siZFAS1 were tested using qRT‐PCR, as shown in Figure 2A. ZFAS1 expression was increased upon transfection with p‐ZFAS1 but suppressed by siZFAS1 (*P* < .01). The CCK‐8 assay (Figure 2B) and colony formation assay (Figure 2C) demonstrated that upregulation of ZFAS1 significantly facilitated the proliferation of HONE1 cells in vitro and that downregulation of ZFAS1 markedly inhibited HONE1 proliferation (*P* < .01). Additionally, a transwell assay was used to determine whether the aberrant expression of ZFAS1 influenced the migratory and invasive abilities of NPC cells. We found both the migration (Figure 2D) and invasion (Figure 2E) of NPC cells were promoted by the upregulation of ZFAS1 and suppressed by the downregulation of ZFAS1 (*P* < .01).

**Figure 2:** LncRNA ZFAS1 enhances the proliferative, colony‐forming, migratory and invasive abilities of NPC cells in vitro*.* A, Expression of ZFAS1 was changed in HONE1 cells transfected with pcDNA3.1‐ZFAS1 (p‐ZFAS1) or ZFAS1‐targeting siRNA (siZFAS1). Transfection with p‐ZFAS1 promoted but transfection with siZFAS1 suppressed the expression of ZFAS1 in vitro. B, CCK‐8 assay showed that ZFAS1 promoted the proliferation of HONE1 cells in vitro. Values of optical density were measured at 450 nm using a plate reader. *P < .01 compared with the NC group by two‐way ANOVA followed by Bonferroni post‐tests. C, Colony formation assay showed that lnc‐ZFAS1 promoted the colony‐forming ability of HONE1 cells in vitro. Cell colonies were visualized and counted using crystal violet staining. D‐E, Transwell assay showed that ZFAS1 promoted the migratory and invasive abilities of HONE1 cells. Cells in the bottom chamber were visualized and counted using crystal violet staining. **P < .01 compared with the NC group

### 3.3 ZFAS1 is necessary for the growth of NPC tumours in vivo

To investigate whether the ZFAS1 is necessary for the growth of NPC tumours in vivo, a xenograft nude mouse model was established. As shown in Figure 3A, the in vivo growth of tumour xenografts formed by shZFAS1‐transfected HONE1 cells was significantly slower than that of tumours formed by HONE1 cells transfected with non‐targeting shRNA (shNC). However, tumour xenograft p‐ZFAS1‐transfected HONE1 cells grew significantly faster than the other two types of cells. After implantation for 21 days, all animals were killed; xenografts were harvested, imaged and weighed. Both the volume and weight of tumour xenografts formed by shZFAS1‐transfected HONE1 cells were significantly decreased compared with those formed by shNC‐transfected HONE1 cells but those of tumour xenografts formed by p‐ZFAS1‐transfected HONE1 cells were significantly increased (Figure 3A‐C, *P* < .01). Then, the expression of ZFAS1 in the tumour xenografts was measured using qRT‐PCR, and the results are shown in Figure 3D. ZFAS1 was obviously down‐regulated in the tumour xenografts formed by shZFAS1‐transfected HONE1 cells but up‐regulated in the tumour xenografts formed by pZFAS1‐transfected HONE1 cells (Figure 3D, *P* < .01). In conclusion, ZFAS1 is necessary for the in vivo tumorigenesis of NPC.

**Figure 3:** LncRNA ZFAS1 promotes tumour formation in nude mice. A, Growth curve of the tumour xenograft formed by HONE1 cells in nude mice. HONE1 cells were pre‐transfected with ZFAS1‐targeting shRNA (shZFAS1) or p‐ZFAS1, and tumour volumes were measured every 3 days. *P < .01 compared with the NC group by two‐way ANOVA followed by Bonferroni post‐tests. Scale bar: 1 cm. B, Schematic representation of tumour xenografts. Animals were killed after implantation for 21 days, and tumour xenografts were harvested and imaged. C, Weight comparison of the harvested tumour xenografts. D, Expression level of ZFAS1 in the xenografts. *P < .05, **P < .01 and ***P < .001

### 3.4 ZFAS1 directly targets miR‐892b

The downstream miRNAs that can be targeted by ZFAS1 were identified by using the miRcode v11 web server. MiR‐892b presented the high affinity with ZFAS1, so it was selected for the subsequent studies. Additionally, the predicted binding site with six consecutive complementary nucleotides was shown in Figure 4A. The dual‐luciferase assay showed that miR‐892b mimics could largely suppress the expression of a reporter plasmid carrying the wild‐type 3’‐UTR sequence of ZFAS1 (*P* < .01), but not the mutant sequence (*P* > .05) (Figure 4B). In addition, compared with that in para‐carcinoma tissues, the expression of miR‐892b in NPC tumour tissues was significantly decreased (*P* < .01, Figure 4C) and was negatively correlated with the expression of ZFAS1 (Figure 4D). In HONE1 cells, the overexpression of ZFAS1 induced by p‐ZFAS1 transfection significantly reduced the expression of miR‐892b, but silencing ZFAS1 induced by siZFAS1 transfection obviously up‐regulated miR‐892b expression (*P* < .01, Figure 4E).

**Figure 4:** The miRNA target of ZFAS1 is miR‐892b. A, Predicted binding sites of miR‐892b on the ZFAS1 transcript. LncRNA‐miRNA interaction was predicted by the miRcode v11 web server. B, Dual‐luciferase reporter assay demonstrated that miR‐892b can target the wild‐type 3’‐UTR of ZFAS1 and significantly inhibit the expression of ZFAS1. Here, miR‐892b mimics or mimics control were separately transfected into HEK293T cells with pmirGLO‐ZFAS1 (wild‐type) or pmirGLO‐ZFAS1 (mutant). **P < .01 compared with cells cotransfected with pmirGLO‐ZFAS1 (wild‐type) and mimics control. C, Comparison of the relative expression of miR‐892b between NPC tissues and para‐carcinoma tissues. **P < .01. D, The expression of miR‐892b in NPC tumour tissues was negatively correlated with expression of ZFAS1. E, Expression of miR‐892b in HONE1 cells was negatively regulated by ZFAS1. **P < .01 compared with HONE1 cells transfected with empty pcDNA3.1 plasmid (NC group)

### 3.5 MiR‐892b inhibits the proliferation, migration and invasion of HONE1 cells in vitro

HONE1 cells were divided into four groups based on transfections with mimics control, miR‐892b inhibitor, miR‐892b mimic or cotransfection with siZFAS1 and miR‐892b inhibitor, and qRT‐PCR was used to test the transfection effects. Compared with cells transfected with the mimic control, miR‐892b mimic transfection group showed higher expression of miR‐892b expression while miR‐892b inhibitor caused the lower expression of miR‐892b (*P* < .01, Figure 5A). Both the CCK‐8 assay (Figure 5B) and colony formation assay (Figure 5C) showed that overexpression of miR‐892b significantly inhibited the proliferation of HONE1 cells and silencing of miR‐892b facilitated the proliferation of HONE1 cells in vitro (*P* < .01). Furthermore, a transwell assay was carried out to detect the migratory and invasive abilities of HONE1 cells with dysregulated miR‐892b expression in vitro. Both the migration (Figure 5D) and invasion (Figure 5E) of HONE1 cells were repressed by the upregulation of miR‐892b and enhanced by the downregulation of miR‐892b (*P* < .01, Figure 5D‐E). Cotransfection of miR‐892b inhibitor and siZFAS1 did not change the expression of miR‐892b and thus failed to influence the in vitro proliferation, migration and invasion of HONE1 cells.

**Figure 5:** miR‐892b inhibits NPC cell proliferation, colony formation, migration and invasion in vitro*.* A, Expression of miR‐892b in HONE1 cells with transient transfection of miR‐892b mimics, miR‐892b inhibitor, siZFAS1 + miR‐892b inhibitor. Transfection of miR‐892b mimics promoted the expression of miR‐892b but transfection of miR‐892b inhibitor suppressed the expression of miR‐892b in vitro. B, CCK‐8 assay showed that miR‐982b suppressed the proliferation of HONE1 cells in vitro. Values of optical density were measured at 450 nm using a plate reader. *P < .01 compared with NC group by two‐way ANOVA followed by Bonferroni post‐tests. C, Colony formation assay showed that miR‐982b suppressed the colony‐forming ability of HONE1 cells in vitro. Cell colonies were visualized and counted using crystal violet staining. D‐E, Transwell assays showed that miR‐982b suppressed the migration and invasion ability of HONE1 cells. Cells in the bottom chamber were visualized and counted using crystal violet staining. **P < .01 compared with HONE1 cells transfected with empty pcDNA3.1 plasmid (NC group)

### 3.6 LPAR1 is the downstream effector of miR‐892b

The downstream mRNA targets of miR‐892b were screened by TargetScanHuman v7.2 web server, and the 3’‐UTR of LPAR1 was selected as a promising target for miR‐892b due to the high affinity between them. Here, two possible binding sites with the same sequence (5’‐AGCCAGU‐3’) were shown in Figure 6A. The dual‐luciferase assay indicated that miR‐892b mimics could largely suppress the expression of the reporter plasmid carrying the wild‐type 3’‐UTR sequence of LPAR1, even if merely bounded to the predicted sites‐1 or site‐2 (*P* < .01, Figure 6B‐C). The expression of LPAR1 was significantly increased in NPC tumour tissues compared with the matching para‐carcinoma tissues (*P* < .01, Figure 6D). Additionally, in Figure 6E, we found that expression of LPAR1 had a significant negative correlation with the expression of miR‐892b in NPC tumour tissues (Figure 6E). In addition, the expression of LPAR1 was positively correlated with the expression of ZFAS1 (Figure 6F). In HONE1 cells, both the expression of LAPR1 mRNA (Figure 6G) and protein (Figure 6H) were largely promoted by transfection with miR‐892b inhibitor but down‐regulated by miR‐892b mimics (*P* < .01). Cotransfection of miR‐892b inhibitor and siZFAS1 did not change the expression of miR‐892b and thus failed to regulate the expression of LPAR1. Furthermore, compared with the NC group, the LPAR1‐targeting siRNA group showed lower expression of LPAR1 (*P* < .01, Figure 7A). Both the CCK‐8 assay (Figure 7B) and colony formation assay (Figure 7C) showed that silencing LPAR1 reduced the proliferation of HONE1 cells in vitro (*P* < .01). Whether LPAR1 affected the migration and invasion of HONE1 cells was also tested using a transwell assay (Figure 7D). Both the migration (top) and invasion (bottom) of HONE1 cells were repressed by the transfection of LPAR1‐targeting siRNA (*P* < .01).

**Figure 6:** The downstream effector of miR‐892b is LPAR1. A, Predicted binding sites of miR‐892b on the LPAR1 transcript. The miRNA‐mRNA interaction was constructed by the TargetScanHuman v7.2 web server. Two binding sites with the same sequences were discovered and designated site one and site two. B, Dual‐luciferase reporter assay was used to verify the predicted binding site‐1 of miR‐892b on the LPAR1 transcript. A partial sequence of LPAR1 3’‐UTR (located at 440‐846, containing the predicted binding site‐1) was cloned into the pmirGLO reporter vector. **P < .01 between transfection with miR‐892b mimics and mimics control. C, Dual‐luciferase reporter assay was used to verify the predicted binding site‐2 of miR‐892b on the LPAR1 transcript. A partial sequence of LPAR1 3’‐UTR (located at 1137‐1609, containing the predicted binding site‐2) was constructed into the pmirGLO reporter vector. **P < .01 between miR‐892b mimics and mimics control. D, Comparison of the relative expression of LPAR1 mRNA between NPC tissues and para‐carcinoma tissues. **P < .01. E‐F, The expression of LPAR1 had a significant negative correlation with the expression of miR‐892b in NPC tumour tissues while the expression of LPAR1 was positively correlated with the expression of ZFAS1. G‐H, Both mRNA and protein expression of LPAR1 in HONE1 cells were negatively regulated by miR‐892b. mRNA expression was detected by qRT‐PCR, and protein expression was detected by Western blot. **P < .01 compared with HONE1 cells transfected with mimics control (NC group)

**Figure 7:** Si‐LPAR1 inhibits NPC cell proliferation, colony formation, migration and invasion in vitro*.* A, Expression of LPAR1 in HONE1 cells transiently transfected with si‐LPAR1. Transfection with si‐LPAR1 suppressed the expression of si‐LPAR1 in vitro. B, CCK‐8 assay showed that si‐LPAR1 suppressed the proliferation of HONE1 cells in vitro. Values of optical density were measured at 450 nm using a plate reader. *P < .01 compared with the NC group by two‐way ANOVA followed by Bonferroni post‐tests. C, Colony formation assay showed that si‐LPAR1 suppressed the colony‐forming ability of HONE1 cells in vitro. Cell colonies were visualized and counted using crystal violet staining. D, Transwell assays showed that si‐LPAR1 suppressed the migration and invasion ability of HONE1 cells. Cells in the bottom chamber were visualized and counted using crystal violet staining. **P < .01 compared with the NC group

## 4 DISCUSSION

Here, we determined the expression profile of lncRNAs in the tumour tissues of NPC patients. The results from the microarray analysis showed that multiple lncRNAs including LINC01000, ZFAS1, APTR, SNHG25, IGHG1 and PP14571 were up‐regulated. However, these lncRNAs were not significantly different between NPC tissues and the para‐carcinoma tissues in the published lncRNA microarray results reported by Zhang, *et al*.^35^ To verify the reliability of our results, qRT‐PCR with a larger sample size (n = 53) was used. Unexpectedly, the expression level of ZFAS1 in a portion in NPC specimens was lower than the average expression level of para‐carcinoma specimens. Thus, we hypothesized that the difference between our results largely resulted from the sample selection for microarray analysis. Overexpression of ZFAS1 has been found to significantly promote the proliferation and inhibit the apoptosis of gastric cancer cells by repressing KLF2 and NKD2 expression.^36^ Additionally, by sponging miR‐150‐5p and thus up‐regulating the expression of transcription factor Sp1 (specificity protein 1), ZFAS1 enhances the proliferative and migratory activities of ovarian cancer cells.^37^ Similarly, ZFAS1 promotes tumorigenesis and metastasis of osteosarcoma through sponging miR‐486.^38^ However, some researchers have considered ZFAS1 as a tumour suppressor for breast cancer.^39^ Here, we found that the high‐expression of ZFAS1 was significantly associated with the T stage (*P* = .0281) and TNM stage (*P* = .0281) in NPC patients. Subsequent studies showed that overexpression of ZFAS1 facilitated the proliferation, migration and invasion of NPC cells as well as the tumorigenesis in nude mice. Chen, *et al* 20 found overexpression of ZFAS1 in NPC tissues and showed that the up‐regulated ZFAS1 could promote the progression of NPC through activation of the Wnt/β‐catenin pathway. Here, we observed another potential mechanism for the tumour‐promoting effect of ZFAS1 mediated by sponging miR‐892b to promote the expression of LPAR1.

In addition to directly regulating the expression of target genes at the epigenetic level, such as the direct repression of KLF2 and NKD2,^36^ lncRNA ZFAS1 also regulates gene expression by acting as an endogenous sponge of miRNAs to inhibit the activity of miRNAs.^40^ For example, ZFAS1 negatively regulates miR‐150 and thus promotes the expression of C‐reactive protein in rats with acute myocardial infarction 41; ZFAS1 overexpression promotes tumour metastasis in hepatocellular carcinoma by releasing the miR‐150‐mediated suppression ZEB1, MMP 14 and MMP 16.^19^ Here, we found that ZFAS1 could indirectly regulate the expression of downstream LPAR1 in a miR‐892b‐dependent manner. Dysregulated expression of miR‐892b has been found to be associated with several diseases including cancer, although the findings are controversial. For example, the increased expression of miR‐892b has been implicated in the development of postherpetic neuralgia,^42^ T2DM‐associated microvascular complications 43 as well as non‐small cell lung cancer.^44^ In colorectal cancer, both the upregulation 45 and downregulation 46 of miR‐892b have been reported. In breast cancer, miR‐892b is significantly down‐regulated in tumour specimens and is closely associated with the poor survival of patients, and silencing of miR‐892b can activate the NE‐κB pathway and promote breast cancer aggressiveness.^25^ Here, miR‐892b was down‐regulated in NPC tissues, which was negatively associated with the proliferative, migratory and invasive abilities of NPC cells. Down‐regulated expression of miR‐892b has also been reported by Xu, *et al*,^26^ who analysed the plasma levels of miRNAs and found that miR‐892b was significantly decreased in NPC patients as compared to healthy controls, but miR‐892b was up‐regulated after treatment with radiotherapy and/or chemotherapy and down‐regulated again when NPC recurred and metastasized. However, although the dysregulated expression of miR‐892b has been reported in the abovementioned diseases, to the best of our knowledge, the upstream regulator of miR‐892b expression so far has been largely unknown. In our present study, the downregulation of miR‐892b in NPC specimens corresponded to the upregulation of ZFAS1. A dual‐luciferase reporter assay verified that miR‐892b could bind to the 3’‐UTR of ZFAS1, while siZFAS1‐induced silencing of ZFAS1 resulted in increased expression of miR‐892b. Therefore, this study provided a promising regulator of miR‐892b expression but whether the dysregulated expression of miR‐892b in other diseases is also caused by ZFAS1 still requires further investigation.

To the best of our knowledge, miR‐892b can mediate the progression of cancers via regulating the expression of pathways such as NF‐κB (breast cancer),^25^ p19ARF/cyclin D1/CDK6 and Sp‐1/MMP‐9 (bladder cancer).^24^ However, how miR‐892b exerts its inhibitory effects on NPC remains unknown. Here, we identified a promising downstream effector of miR‐892b in NPC as LPAR1. The expression of LPAR1 in NPC cells was negatively regulated by miR‐892b. LPA is a small phospholipid molecule that promotes cancer progression and metastasis, and aberrant regulation of the LPA signalling pathway may be caused by an increase in LPA synthesis, thus changing the profile of circulating LPA and causing dysregulation of LPAR.^47^ Blockage of LPA receptors using pharmacological methods (eg BrP‐LPA, a pan‐LPA antagonist) significantly inhibited the in vitro motility of human breast cancer cell MDA‐MB‐231.^48^ Among these LPARs, LPAR1 is up‐regulated and exhibits pro‐oncogenic and pro‐metastatic properties in various primary tumours including breast cancer, hepatic cancer and ovarian cancer.^49^ Regarding NPC, expression of LPAR1 mRNA in NPC specimens was significantly higher than that in noncancerous specimens. LPAR1 silencing by transfection with miR‐892b mimic or LPAR1‐targeting siRNA significantly inhibited the invasion of NPC cells in vitro. Although, we found that LPAR1 could act as the main mediator responsible for LPA‐stimulated ovarian cancer cell invasion in other studies,^29^, ^50^ there had been no previous studies focusing on the effect of LPAR1 regulating nasopharyngeal carcinoma. Therefore, we chose LPAR1 as target for miR‐892b.

Overall, the expression of lncRNA ZFAS1 was significantly elevated in NPC tissues and cells, which had important implications for the tumorigenesis and metastasis in NPC. Down‐regulated expression of lncRNA ZFAS1 was sufficient to inhibit the proliferation, migration, invasion of NPC cells in vitro and tumorigenesis in vivo. The cancer‐promoting activity of ZFAS1 mainly depended on its sponging effect to miR‐892b and the subsequent upregulation of LPAR1, but whether the dysregulation of miR‐892b and LPAR1 is only mediated by the upregulation of ZFAS1 still needs future study to illustrate.

## CONFLICTS OF INTEREST

The authors confirm that there are no conflicts of interest.

## AUTHOR CONTRIBUTIONS

JJP, FL and HZ performed the research; JJP, QW and SXL designed the research study; JJP, FL, HZ and QW analysed and interpretation the data; JJP and SXL wrote the paper; SXL revising it critically; all authors approved the submission of final versions.

## ETHIC APPROVAL AND INFORM CONSENT

The research was carried out according to the World Medical Association Declaration of Helsinki and approved by West China Hospital, Sichuan University. Written informed consents were obtained from all participants.

## Data Availability

The data that support the findings of this study are available from the corresponding author upon reasonable request.
